# Upper Arm Motion High-Density sEMG Recognition Optimization Based on Spatial and Time-Frequency Domain Features

**DOI:** 10.1155/2019/3958029

**Published:** 2019-03-25

**Authors:** Dianchun Bai, Shutian Chen, Junyou Yang

**Affiliations:** School of Electrical Engineering, Shenyang University of Technology, Shenyang 110870, China

## Abstract

**Background:**

Spatial characteristics of sEMG signals are obtained by high-density matrix sEMG electrodes for further complex upper arm movement classification. Multiple electrode channels of the high-density sEMG acquisition device aggravate the burden of the microprocessor and deteriorate control system's real-time performance at the same time. A shoulder motion recognition optimization method based on the maximizing mutual information from multiclass CSP selected spatial feature channels and wavelet packet features extraction is proposed in this study.

**Results:**

The relationship between the number of channels and recognition rate is obtained by the recognition optimization method. The original 64 electrodes channels are reduced to only 4-5 active signal channels with the accuracy over 92%.

**Conclusion:**

The shoulder motion recognition optimization method is combined with the spatial-domain and time-frequency-domain features. In addition, the spatial feature channel selection is independent of feature extraction and classification algorithm. Therefore, it is more convenient to use less channels to achieve the desired classification accuracy.

## 1. Introduction

Analysis of user's intention through noninvasive surface electromyography acquisition methods has the advantages of shorter experimental preparation time and more convenient acquisition. Noninvasive sEMG analysis has been widely used in prosthesis [1, 2], exoskeleton [3], and rehabilitation robot control [4–6]. Pattern recognition based on EMG signal processing was adopted by growing smart prosthetic hands and arms control [7–9]. Rd [10] achieved the hand motion classification by analyzing time-domain features of the EMG signal. In addition, Hudgins et al. [11] used the frequency-domain and time-frequency-domain features analysis method to obtain a desired classification result for the specific actions based on EMG signals. In these methods, few electrodes (<16 channels) were used for recording EMG signals, which are arduous to obtain the most active muscle positions channels. Electrodes were shifted during each experiment. An uncertainty shifted electrode position caused worse classification results. Moreover, few electrodes provide insufficient sEMG features, which decline complex movement classification accuracy [12]. Studies [13] showed that when a person does some movements, the active muscles do not contract simultaneously. Ordinarily, muscle contraction causes joint motion and a group of muscles contraction are ahead of others. sEMG signals information amplitude from the monopolar electrode is relevant to the electrode position, and if the electrode recording position deviates from the main contraction areas, signal amplitude will be lower. In addition, when the electrodes need to be replaced, the electrode position would be shifted and then the sEMG signal recorded at the original electrode position is accompanied by an unpredictable change, which leads to an obvious classification accuracy reduction. The solution is to retrain the classifier. Otherwise, the electrode shift or offset will deteriorate EMG control robustness and pattern recognition reliability.

Recently, the two-dimensional high-density electrode sEMG signals acquisition technique has been used in pattern recognition analysis [14]. The high-density surface electromyography analysis method is a noninvasive technique with multiple electrodes that can measure electrical activity of muscles in the limited area of skin and capture temporal and spatial information in the whole muscles EMG activation region. Using high-density acquisition electrodes device can not only overcome the shortcomings of the poor robustness of the monopolar electrode shifted but also can detect some small movements of muscles activity signal information. In addition, more sEMG acquisition channel electrodes are used to achieve better motion classification performance, which is beneficial to prosthetic arm control [15]. At the same time, the topographic map of activity signals amplitude intensity of the high-density electrode matrix analysis method is used to determine the electrode position of the region where the muscles motion potential activity is relatively strong [16, 17]. Vieira et al. [18] used the segmentation recognition method for the active region of high-density EMG signals to extract the EMG signals features on the muscle activation region and to improve the accuracy and robustness of the pattern recognition classifier. However, the increasement of high-density signal electrode channels aggravated data processing burden. EMG signals were collected from the channels of high-density matrix electrodes, containing large amounts of artifacts and redundant information, while processing these data would make classifier overfitting and reduce classifier's recognition accuracy. Therefore, separating the useless information and reducing the processing amount of the data are beneficial to improve the pattern recognition [19]. The spatial filtering algorithms principle component analysis (PCA), independent component analysis (ICA), and common spatial pattern (CSP) [20] are carried out by using the 128-channel EEG signals [21] for spatial-domain feature extraction. The original signal components were extracted from the original signals. It will reduce the computational dimension of the original data and the amount of data processing.

To extract more features of each sEMG signal channel, the method is proposed by gathering time-domain and frequency-domain signal characteristics from the selected high-density signal channels. Performance and practicality of the algorithm will be enhanced by selecting more channels of active signal characteristics, and this paper focuses on selecting more active channels automatically and gathering useful information from these channels. Wang et al. [22] used the wavelet packet transforms to extract the time-frequency domain characteristics of the active EMG signals, which were collected by 46 high-density matrix electrodes. The analytical methods that combined Fisher's class separability index with sequential feed forward selection were used for selecting the characteristics channels. The average classification accuracy was 98.53% when 46 channels were selected; when 10 predetermined channels were selected, the accuracy rate reached 92.92%. The disadvantage of this method is that all channels EMG decomposed by the wavelet packet will produce higher dimension data, which leads to huge data calculation. Moreover, this algorithm of channel selection largely relies on EMG features and classification algorithms. Geng et al. [23] applied the one-versus-rest (O*v*R) scheme to multiclass CSP channel selection algorithms. Firstly, 56-channel high-density matrix electrodes were used to acquire signals. Secondly, time-domain characteristics were extracted for the selected channel. Finally, motion classification by the LDA and KNN classification algorithm is employed, average classification accuracy rate is 94.5% when 56 channels were selected, and if 18 channels are used, the accuracy rate is 93.3%. The advantage of this method is that the channel selection algorithm is independent of the feature extraction and classification algorithm, when the feature and classification algorithm need to be changed, channel selection becomes more convenient, and the dimensionality problem of high-dimension feature need not be considered. Its disadvantage is that it still needs more channels to achieve the desired classification accuracy.

In this work, the multiclass CSP algorithm was adopted by joint approximate diagonalization (JAD) [24] as the data preprocessing method. A spatial feature channel selection method was proposed to select the less channels based on maximize mutual information for different types of the sEMG signal, and the feature extraction method of the wavelet packet transform (WPT) was used to extract wavelet coefficients characteristics for different frequency bands of EMG data of the selected channels. Finally, pattern recognition was realized by the SVM classification algorithm. There are two purposes of the proposal idea. First, channel selection is for the next feature extraction and pattern classification algorithm. Second, WPT is for achieving feature segmentation of the EMG signal from the selected channel. Finally, the method will achieve the desired classification accuracy by selecting fewer channels.

In this paper, high-density sEMG provides important guidance for optimizing the electrode number and location to detect the intended movements. The structure of the shoulder joint is more complicated. The movement of the upper arm activates the muscle group and causes the upper arm to perform various movement modes. When upper arm does different movements, it often needs more muscles to coordinate [25]. Upper arm EMG signal resolution is difficult to obtain, accuracy rate of pattern recognition is low, Naik et al. [26] used the HD-sEMG signal for optimal muscle selection, it indicates that it is not necessary to perform all muscle signal analysis, and only the muscles close to the wrist can be used to resolve the soft movement of the fingers. At the same time, it is verified by the optimization algorithm and shoulder motion analysis of the muscles coordinated motion. Furthermore, the upper arm EMG analysis will benefit for prosthetic arm control for patients with high upper limb amputations.

The following is organized in three sections. The next section describes the methods of high-density surface EMG recording and myoelectric pattern recognition.  Section 3 describes the experimental results, followed by the discussions and the conclusion in Section 4.

## 2. Experimental Setup

In this work, three healthy experimental subjects were selected. sEMG signals were recorded by a 64-channel high-density matrix electrode, which is made by OT Bioelectronics in Italy, as shown in Figure 1(a). 64-channel high-density matrix-type electrode arrangement is 5 rows × 13 columns, the spacing between adjacent electrodes is 8 mm, the diameter of each electrode is 3 mm, and the number and position of 64 channels are arranged in a certain order, which is convenient to determine the electrode position by the channel number. In addition, the reference electrode that is like spire lamella is worn on the subject wrist. As showed in Figure 1(b), the high-density surface electrode is placed on the medial deltoid muscles position of the subject's upper arm. The deltoid muscles contract when the upper arm movements [24].

Before the electrodes are pasted, target skin needs to be cleaned by alcohol for reducing skin resistance. Between the skin and electrode, a double-sided electrode sheet coated with conductive gel is used (the electrode sheet is affixed with upper and lower sides; one side is pasted on the subject's skin, and the other side is pasted on the high-density matrix-type electrode sheet, where the electrode hole is coated with a conductive gel to enhance the conductivity) that the skin will be closely adhered to the electrode sheet. The other end of the high-density matrix electrode is connected to the amplification system (EMG-USB2+, OT Bioelectronics, Italy), with a signal magnification of 1000 and a sampling frequency of 5120 Hz.

Before the experiment, each subject sits comfortably on a chair. Then, subjects start to be familiar with the whole process of the experiment. After subjects understand the whole experiment, subjects are scheduled to complete the intended action at the prompt of the sound guide. The experimental process lasted for 50 s. Multiple muscles participate in the body to do certain movement. Maintaining the same posture for a long time can cause muscle fatigue, resulting in muscle compensation. The angle sensor measures the angle of the main force muscle. When experiment starts, the subject's upper arm does the forward flexion and horizontal flexion motion with 8 different kinds of angles. The diagram of the specified motions is shown in Figure 2. Each motion lasts for 2 s and then continues to do the next motion. When the overall motion is completed, subject's take a minute and then start the next experiment to prevent muscles fatigue. Each subjects' experiments are repeated five times. The whole process of EMG data acquisition is completed by the EMG signal recording software (OT Biolab).

## 3. Spatial Filtering Principle and Analysis

High-density matrix electrode is used in this work which contains 64 channels. The recorded signals contain several redundant and artifact signals. To be able to separate the useful signal from original signals, three spatial filtering algorithms CSP, ICA, and PCA are used in data preprocessing. In the three spatial filtering algorithms, raw data are used to calculate the spatial filter matrix *ω*=[*ω*_1_,…, *ω*_*n*_], through which *y*(*t*)=[*y*_1_(*t*),…, *y*_*n*_(*t*)], the principle components of raw data, are obtained. The implementation process uses *W* to multiply the original EMG signal *x*_*t*_ to calculate *y*_*t*_=*W*^*T*^*∗x*(*t*).

### 3.1. Principle Component Analysis

The essence of PCA is to maximize the representation of the original data features as much as possible, the orthogonal transformation of multivariate data to its relevance, and projected onto a new coordinate system such that the largest variance in the data lies on the first coordinate and the smallest variance in the data tends to the last coordinate. PCA is an unsupervised spatial filtering algorithm that is used to determine the number of principal components. That is, if the number of channels for collecting the sEMG number is n, the dimension of the separation matrix is n*∗*n. Raw sEMG signal is processed by the PCA, and the dimension of *W* becomes only *k∗n*(*k* ≤ *n*). As shown in Table 1, the PCA spatial filtering algorithm is used to determine the number of principal elements by the cumulative contribution rate when six subjects have eight different motion angle modes in the shoulder joint. In order to reduce the processing amount of the original sEMG data as much as possible, the average value of each experimenter subjects's sEMG data in eight different action modes is selected as the number of principal elements of the final filter matrix. HD-sEMG signals of the upper arm eight different motions are preprocessed by the PCA spatial filtering algorithm. 64 channels of sEMG data are projected to low-dimensional representation by linear transformation without discarding the original sEMG information features. The subject eight different motion high-density sEMG signal spatial filter preprocessing results by PCA are shown in Figure 3; the linear dimensionality reduction process of the original sEMG data is visualized by PCA and the contribution rate is calculated to be 95%; the separation matrix is determined to retain the least number of spatial filters, which achieves the purpose of reducing the number of dimensions.

### 3.2. Independent Component Analysis

FastICA algorithm extracts independent components from the mixture data, which is an effective method for signal blind source separation. Its fast convergence (secondary convergence at least) is easy-to-use (no need to set the step parameters), which has been widely used in medical signals processing [27]. It is based on the principle of maximum negentropy to analyze the independent components in non-Gaussian mixed signals. Raw signals are averaged and whitened. Then, independent components are extracted. The implement process is to reduce errors accumulation that *n* independent components were processed at the same time using symmetric orthogonal, and *W* is applied to raw data *y*=*W*^*T*^*∗x*, which obtains independent components of *n* channels that removed interference. The visualization is shown in Figure 4.

### 3.3. Spatial Filtering Algorithm of HD-sEMG Based on Multiclass CSP

CSP is a supervised two-class spatial filtering algorithm [21]. Spatial filtering *W* can maximize one class variables while minimizing the other class variables. This method was proposed by Blankertz [28], which has been successfully applied to two categories EEG/MEG data pattern recognition. *X*_1_ and *X*_2_ represent the original signal two categories data matrix (*n∗d*), *d* is the number of signal channels, and *n* is the number of sampling points for each channel signal. The purpose of the algorithm itself is to calculate a filter matrix *W* that maximizes the class 1 variables while minimizing the class 2 variables and is shown in the following equation:

(1) $$\begin{array}{c} W=\arg\max\frac{W^{T}\sum_{1}W}{W^{T}\sum_{2}W}. \end{array}$$

The linear filtering matrix *W* is obtained by solving the problem of a generalized eigenvalue, while diagonalizable simultaneously by the covariance matrix:

(2a) $$\begin{array}{c} W\underset{1}{\sum }W^{T}=D_{1}, \end{array}$$

(2b) $$\begin{array}{c} W\underset{2}{\sum }W^{T}=D_{2}, \end{array}$$

(3) $$\begin{array}{c} D_{1}+D_{2}=I. \end{array}$$

The columns number of the *W* matrix is equal to the number of spatial filters *L*, and application of spatial filtering matrix *W* to raw signal data will be *L*-dimensional output signal, *y*=*W*^*T*^*∗x*, which is principle components of the raw signals.

In addition, there are several methods to extend the CSP algorithm into multiclass paradigms analysis by performing two-class CSP on different combinations of classes. One approach is to combine multiple two-class CSP methods based on one class versus all other class (O*v*R) or one class versus another class (O*v*O) scheme [28] and another method based on joint approximation diagonalization with diagonalizable simultaneously multiclass covariance matrices (JAD) [21]. *W* is obtained by diagonalization covariance matrices of multiclass at the same time, *W*∑_*c*_*i*__*W*^*T*^=*D*_*c*_*i*__, ∑_*c*_*i*__*D*_*c*_*i*__=*I*, *i*=1,…, *M*, is the number of classes.

In this work, the multiclass CSP algorithm is employed in JAD, which spatial filtering matrix *W* is calculated based on different class covariance matrices. The multiclass CSP method was proposed by Grosse *et al.* [21] based on the JAD, which will project the mixture signal into the space where the raw signal is orthogonal to the noise signal. The visualization of covariance matrix ∑_1_,…, ∑_8_ for eight different motions HD-sEMG is shown in Figure 5. The block structure of the covariance matrices is caused by the row-wise positioning of the channels within the electrode arrays.

It can be seen in Figure 5 that the magnitude color change in the visualized covariance matrix that the fast Frobenius diagonalization (FFDIAG) [29] is used in diagonal eight different action covariance matrices, and eight different motion classes diagonalization matrices are *D*_1_,…, *D*_8_. The main diagonal element of Dc is the eigenvalue spectrum from class c. As in the binary case, the eigenvalue *λ*_*i*_^*c*^ indicates the variance of cow component *i* for signals of class *c*.

Selecting specific components for classification is not straightforward as in the binary case, where the component with highest eigenvalue for one class has automatically the lowest eigenvalue for the other class. However, multiple classes of the covariance matrix simultaneously diagonal method are used for specific implementation of the multiclass CSP algorithm. In addition, the number of spatial filtering Cs is chosen as a free parameter in the two-class CSP algorithm. For the two classifications of the problem in [24], the number of Cs was chosen between 2 and 4. However, there is no fixed method for selection of Cs numbers in multiclass CSP algorithms. Para et al. [30] proposed a strategy that assumed two different eigenvalues for the same pattern have the same effect if their ratios to the mean of the eigenvalues of the other classes are multiplicatively inverse to each other, and thus all eigenvalues *λ* are mapped to score (*λ*)=max(*λ*, 1/(1+*N*)^2^*λ*/(1 − *λ*)) and a specified number *m* of highest scores for each class are used as CSP patterns.

### 3.4. Multiclass CSP Filter Number Selection Algorithm Based on Mutual Information Maximization

The multiclass CSP based on the FFDIAG algorithm is used to determine the spatial filter matrix *W* and a method based on maximizing the mutual information between the category *c*, and the reconstruction matrix *W*^*T*^*∗x* is proposed to determine the spatial filter number of the spatial filter matrix. Its purpose is to be able to select the dimensions of the original EMG data. The spatial filter number for spatial filtering matrix *W* of each column is calculated by maximizing the mutual information between class labels *c* and reconstructed signal matrix *ω*^*T*^*x*, shown as follows:

(4) $$\begin{array}{c} \omega^{*}=\arg\max\left\{I\left(c,\omega^{T}x\right)\right\}. \end{array}$$

The mutual information between *c* and *y*=*ω*^*T*^*x* is shown in the following equation:

(5) $$\begin{array}{c} I\left(c,\omega^{T}x\right)=H\left(\omega^{T}x\right)-H\left(\omega^{T}x\left|c\right.\right)=H\left(y\right)-\overset{M}{\underset{i=1}{\sum }}P\left(c_{i}\right)H\left(y\left|c_{i}\right.\right). \end{array}$$

The entropy of *y* given class labels *c*_*i*_ is

(6) $$\begin{array}{c} H\left(y\left|c_{i}\right.\right)=\log\sqrt{2\pi e\sigma_{y\left|c_{i}\right.}^{2}}=\log\sqrt{2\pi e\omega^{T}\underset{c_{i}}{\sum }\omega }. \end{array}$$

The marginal distribution *p*(*y*), however, does not follow a Gaussian distribution:

(7) $$\begin{array}{c} p\left(y\right)=\overset{M}{\underset{i=1}{\sum }}p\left(c_{i}\right)p\left(y\left|c_{i}\right.\right)\sum p\left(c_{i}\right)N\left(0,\sigma_{y\left|c_{i}\right.}\right). \end{array}$$

The definition of negentropy is

(8) $$\begin{array}{c} J\left(y\right)=H_{g}\left(y\right)-H\left(y\right), \end{array}$$

where *H*_*g*_(*y*) is the entropy of the Gaussian random variable with the same as *y* and the negentropy of *y* can be approximated as

(9) $$\begin{array}{c} J\left(y\right)\approx \frac{1}{12}k_{3}{\left(y\right)}^{2}+\frac{1}{48}k_{4}{\left(y\right)}^{2}, \end{array}$$

with the third-order and fourth-order cumulates *k*_3_(*y*)=*E*{*y*^3^} and *k*_4_(*y*)=*E*{*y*^4^} − 3[4]. Since p(y) is the probability density of a sum with a zero mean Gaussian distribution, it is symmetrical. So *k*_3_(*y*)=0. On combining (7) and (8), we obtain the following equation:

(10) $$\begin{array}{c} H\left(y\right)\approx \;\;\log\sqrt{2\pi e-\frac{3}{16}}{\left(\overset{M}{\underset{i=1}{\sum }}p\left(c_{i}\right)\left(\sigma_{y\left|c_{i}\right.}^{4}-1\right)\right)}^{2}, \end{array}$$

where the method of evaluating the mutual information between class *c* and *y* is derived by combining (5), (6), and (10).

(11) $$\begin{array}{c} I\left(c,y\right)\approx -\overset{M}{\underset{i-1}{\sum }}p\left(c_{i}\right)\text{log}\sqrt{W^{T}\underset{c_{i}}{\sum }\omega }-\frac{3}{16}\overset{M}{\underset{i=1}{\sum }}p\left(c_{i}\right){\left({\left(\omega^{T}\underset{c_{i}}{\sum }\omega \right)}^{2}-1\right)}^{2}. \end{array}$$

After the covariance of raw class EMG data is JAD, spatial filtering matrix *W* is obtained by descending the mutual information of each column of *W* by (11). In this work, EMG signals were preprocessed by three spatial filter methods. This purpose is to extract principal components of the raw signal in 64 high-density matrices. Then, the great performance spatial preprocess algorithm will be applied to the upper arm motion classification.

### 3.5. Multiclass CSP Channel Selection Algorithm Based on Mutual Information Maximization

In fact, *W* is constructed by these spatial filtering algorithms and the reconstructed raw signal principal components represent a raw signal to the greatest extent, but raw signal information is lost. It cannot be determined whether it contains the action pattern information. In addition, the principal component is formed by separation matrix *W* reconstruction, if it does not reduce the number of channels which will increase calculation time for subsequent signal processing. However, it is desired that the appropriate number of channels is selected and the electrodes position will be determined, which will be applied to actual prosthetic control. Therefore, the appropriate channel selection algorithm has important application significance. In Grosse's research [22], only extracted *L* columns in spatial filter *W* is extracted to represent spatial subset of raw signal feature information with maximized mutual information and reconstructed to expected principal component *L*-dimensional EMG signal preprocessed matrix *y*. For subsequent pattern recognition, although good results have been achieved, specific method of *L* number selection has not been given. In this work, spatial filtering matrix *W* is used to find the number of raw channels that determine the *L* dimension based on maximizing the mutual information between class *c* and principal component *y*. The less original channel (*L*′ < *L*) EMG data are selected by wavelet packet decomposition analysis, and wavelet coefficients under different frequency segments are extracted, which greatly reduces data processing capacity and calculation time. It not only solves the problem of subject's original EMG motion intention information lost for reconstructing subspace *y* but also reduces the amount of data processed, which will be described below. The 64-channel EMG data preprocessing algorithm of the channel selection process is as shown in Table 2.

## 4. Feature Extraction and Analysis of HD-sEMG

### 4.1. Spatial-Domain Feature Extraction

The HD-sEMG spatial features of the shoulders of the different joints in the upper limb extension and abduction are shown in Figure 6. From this, the characteristic trend of the shoulder joint and the analysis method of the HD-sEMG signal characteristics can be visually obtained. The multiclass CSP channel selection method based on mutual information maximization is proposed in the previous section, the number of channels with strong muscle source signals is selected, and the original sEMG data for the selected signal channel are selected. The WPT method is used to complete the feature subdivision of the frequency domain of the signal; that is, the signal feature is extracted based on the spatial characteristics.

### 4.2. Time- and Frequency-Domain Feature Extraction

Firstly, EMG signals are preprocessed by PCA, FastICA, and multiclass CSP spatial filtering algorithm to obtain the separation matrix *W* which reconstructed EMG data, and then, the different classes are decomposed in detail by WPT, and the logarithm of the RMS value of wavelet coefficients at different frequencies are extracted as the eigenvalue. WPT is an extension of the traditional wavelet decomposition method to provide time-frequency analysis of multiresolution for nonstationary signals, the original signal space as *Ω*_0,0_, and WPT can split signals into an approximation subspace *Ω*_1,0_ and a detail subspace *Ω*_1,1_. Each approximation or detail obtained from the top level, supposed in the subspace *Ω*_*j*,*k*_, will be further split into a new approximation and a new detail, located in two orthogonal subspaces *Ω*_*j*+1,2*k*_ and *Ω*_*j*+1,2*k*+1_. This process will be iteratively performed to a targeted depth *J*. Here, *J* is a scale index ranging from 0 to *J* and *k*  represents subband index with in the scale, ranging from 0 to 2^*J*^ − 1. Consequently, WPT generates a binary tree structure of subspaces spanned by a set of bases, to which a signal will be mapped for multiresolution analysis. Such a characteristic makes WPT to apply in feature extraction successfully. In this paper, the wavelet packet of the fifth order symlet mother wavelet function is used in each channel of the EMG signal, and the number of decomposed layers is *J*=4. Finally, logarithmic RMS of wavelet coefficients of different frequency domains in the *J*^th^ layer composed subsequent pattern classification.

Secondly, the multiclass CSP channel selection method is adopted based on maximizing mutual information according to the spatial feature distribution of HD-sEMG. The optimal number of spatial feature channels is selected, and WPT method is used to select original channels which can maximize the mutual information between different types of channels EMG decomposition in detail; the last layer of wavelet coefficients at different frequencies RMS is extracted as the eigenvalue for pattern recognition. Its advantage is that only the selected channels EMG are decomposed by the wavelet packet will produce less dimension data than with all channels. In addition, it can extract wavelet coefficients characteristics for different frequency bands EMG data.  Figure 7 shows scatter distribution of sEMG time-frequency feature by WPT that is processed by three spatial filtering algorithms obtained.

### 4.3. Analysis of HD-sEMG Spatial-Domain and Time-Frequency-Domain Features

For the spatial feature distribution of HD-sEMG, based on the multiclass CSP channel selection method of maximizing mutual information, the spatial channel with strong spatial distribution of the source signal is selected, and the WPT method is used to maximize the mutual information between different types of channels. The original channel sEMG is decomposed in detail, and the RMS of the wavelet coefficients decomposed into the fourth layer at different frequencies is obtained as the target action to generate the eigenvalues of the HD-sEMG signal for the subsequent pattern classification. As shown in Figure 8, it can be seen from the distribution of feature scatters in 3D and 2D space that the hierarchical clustering effect of feature points in each category is obvious. The feature extraction method can greatly reduce the processing amount of the HD-sEMG signal while effectively extracting the signal characteristics and has the advantage of small data processing amount and is suitable for the analysis of the HD-sEMG signal.

## 5. Pattern Recognition

In this work, different numbers of principal components are selected by the FastICA algorithm, and the classification accuracy of four classifiers is compared, as shown in Figure 9. When different numbers of ICs are selected, classification accuracy of four classifiers will be compared. PCA is used to analyze the principal component channels data at eight different motion patterns, and original 64-channel signals are transformed into linearly independent. The 12-dimensional filters are obtained with the 95% contribution rate for original data. It will reduce the dimension of the preprocessing matrix. 64-channel EMG signal data for eight different motions classification analysis of the experiment are carried out by PCA, in which 12-dimensional EMG data were obtained. PCA are also used to determine the number of ICs for the FastICA, which will resolve the problem to determine the number of ICs by FastICA.

The covariance matrix of the EMG signals is calculated for the eight different motions by the multiclass CSP algorithm. Then, the reconstructed EMG signal dataset time-frequency domain feature was extracted. When the numbers of selected spatial filters are different, the classification accuracy of each classifier is shown in Figure 10. It demonstrates that the number of spatial filters ICs is chosen between 12 and 15, which in case of 16 Cs, is chosen. Reconstructed EMG signals for eight different motions with time-frequency domain feature are analyzed; four classifiers achieve high classification accuracy.

Original channels were selected by the maximized mutual information multiclass CSP algorithm in Figure 11, which was compared with the reconstructed signal methods based on the spatial filter matrix by multiclass CSP for the eight different movements. Apparently, if the five channels were selected, the accuracy of the classifier LDA, SVM, and KNN must exceed 80%, where the accuracy of SVM is 94.3%, which is 5.7% higher than the classification accuracy of SVM when selecting Cs = 12 as the reconstructed EMG signal. It manifests a favorable classification performance by this method. When the number of selected channels is more than 10 channels, the recognition rates of the four classifiers are higher than 80%, and the recognition rates of LDA, SVM, and KNN are 91.3%, 95.1%, and 89.9%, respectively. Therefore, it is concluded that the multiclass CSP algorithm with maximum mutual information is superior to motion pattern recognition based on extraction of a few channel data of the original EMG signals.

The 2D plots scatter diagram is composed of column1 and column2 eigenvalues in Figure 12 that the multiclass CSP algorithm selects the training and prediction results of the fivefold cross validation of the top 16 electrode channel characteristic matrix datasets of the eight different motion angles when the mutual information between the class labels and the different components is maximization. It can be seen from Figure 12 that the processed data features have good separability.

In this work, different spatial filtering algorithms are used to extract the principal components which are PCA, FastICA, and multiclass CSP. They are based on mutual information maximized channel selection for the upper arm eight different motion degrees EMG data (when the number of spatial filters was ICs = 12 and Cs = 12), and pattern recognition results of the four classifiers are shown in Figure 13. When the first five original EMG channels are selected based on the different types of mutual information maximization methods, eight different motions of sEMG data were preprocessed by the four spatial filters, which are applied to the four classifiers ANN, SVM, LDA, and KNN. The accuracy of combination CSP + WPT + SVM (95.1%) and the recognition accuracy rate of SVM are superior to LDA, KNN, and ANN. The confusion matrix plot for eight different motions by the SVM classifier is as shown in Figure 14. The rows show the true class, and the columns show the predicted class. The diagonal cells show where the true class and predicted class match. If these cells are green, the classifier has performed well and classified observations of this true class correctly.

The classification accuracy of the first three motions is 100%, and the fourth to eighth motions are, respectively, 94%, 88%, 97%, 97%, and 85%. It can be seen from Figure 8 that the first three motions feature points are distinguishable. However, the fourth to the eighth motion feature points are densely distributed, and there are more overlapping points; therefore, the classification accuracy of the latter five motions is slightly lower.

It is concluded that a better way to solve the problem of HD-sEMG pattern recognition by multiclass CSP based on mutual information maximization using multiclass CSP + WPT + SVM. At the same time, the original sEMG is selected by maximizing mutual information. If 4-5 optimal channels are selected, accuracy rate reaches to 92%, and amounts of processed channels is less than 10% than the original channels. It is suitable for the EMG prosthesis arm control.

## 6. Conclusion

In this work, 64-channel HD-sEMG technique was used to evaluate the myoelectric signal pattern recognition for the upper arm forward flexion and horizontal flexion motion by analyzing the spatial- and time-frequency-domain sEMG signals characteristics. High-density matrix electrodes introduce large data processing problems to the processor. Therefore, a recognition optimization method is proposed based on the combination of the maximum mutual information channel selection, wavelet packet feature extraction, and support vector machine (SVM) by using the high-density electrode sEMG signal acquisition device, which is, respectively, compared with three spatial filtering (PCA, ICA, and CSP). Four classifications ANN, SVM, LDA, and KNN are used, which are suitable for EMG pattern recognition. When performing this kind of movement recognition, the original 64 electrodes will be reduced to only 4-5 active signal channels and obtain more than 92% accuracy at the same time. The performance of the classifier was analyzed by selecting the number of principal components for the three kinds of spatial filtering algorithms. The PCA algorithm is used to determine the number of ICs.

## Figures and Tables

**Figure 1:** Experimental diagram of 64-channel high-density matrix electrode acquisition: (a) 64-channel (5 rows × 13 columns) high-density matrix-type electrodes and number and position of each channel; (b) high-density surface electrodes' position on the subject's medial deltoid muscles of the upper arm.

**Figure 2:** Diagram of the subject's upper arm motion pattern.

**Figure 3:** High-density sEMG data of subject's eight different motion modes spatial filtering by PCA. (a)–(h) Eight different motions using high-density sEMG data projection of the three-dimensional visualization scatter map by PCA; (i)–(p) eight different of motion high-density sEMG data projection cumulative contribution rate chart by PCA.

**Figure 4:** The diagram of independent components of HD-sEMG data in eight different motions by FastICA.

**Figure 5:** Visualization of covariance matrix data for eight different motions HD-sEMG.

**Figure 6:** High-density sEMG spatial map of eight different degrees when the subject's shoulder extended and abducted motion.

**Figure 7:** Scatter distribution of HD-sEMG in eight different motions of the shoulder extracted from RMS features after WPT decomposition by three different spatial filtering algorithms: (a) scatter distribution of RMS by WPT for raw HD-sEMG signals; (b) scatter distribution of RMS by WPT for the reconstructed sEMG signals by PCA; (c) scatter distribution of RMS by WPT for the reconstructed sEMG signals by FastICA; (d) scatter distribution of RMS by WPT for the reconstructed sEMG signals by multiclass CSP.

**Figure 8:** Scatter distribution of RMS by WPT after channel selection based on mutual information maximization multiclass CSP.

**Figure 9:** Average classification accuracy of four recognition algorithms in the selection of different ICs by FastICA.

**Figure 10:** Average classification accuracy of four recognition algorithms in the selection of different Cs by multiclass CSP.

**Figure 11:** Average classification accuracy of four recognition algorithms when the number of different channels is selected with the mutual information from the high to low order.

**Figure 12:** Scatter diagram of training and testing results between features dataset columns 1 and 2 with the maximum mutual information of the 16 channels by the SVM classifier algorithm: (a) scatter diagram between column 1 and column 2 of original time-frequency features dataset; (b) scatter diagram between column 1 and column 2 of the results of SVM classifier prediction.

**Figure 13:** Four different classifiers average recognition results by using a different combination spatial filtering algorithm.

**Figure 14:** The confusion matrix plot for eight different motions by the SVM classifier.

**Table 1:** Different experimenter subjects in eight different motions using PCA spatial filter through the cumulative contribution rate to determine the number of principle component.

Select PCs	Mode 1	Mode 2	Mode 3	Mode 4	Mode 5	Mode 6	Mode 7	Mode 8	Average value
Subject 1	36	22	6	4	5	7	6	6	12
Subject 2	36	22	6	4	7	7	6	6	12
Subject 3	28	13	5	4	7	7	6	6	10
Subject 4	30	12	5	4	7	7	6	6	10
Subject 5	32	17	6	4	7	7	6	6	11
Subject 6	28	21	6	4	6	7	6	6	11

**Table 2:** Spatial feature extraction based on multiclass CSP.

*Input*: covariance matrices ∑_*x*|*c*_*i*__, *i*=1,…, *M*
(1) Perform joint approximate diagonalization s.t.*w*^*T*^∑_*x*|*c*_*i*__*w*=*D*_*c*_*i*__, *i*=1,…, *M*
(2) For each column *w*_*j*_, *j*=1,…, *N*, of *w* scale *w*_*j*_s.t.*w*_*j*_^*T*^∑*w*_*j*_=1, estimate mutual information according to $I\left(c,y\right)\approx -\sum_{i=1}^{M}p\left(c_{i}\right)\log\sqrt{W^{T}\sum_{c_{i}}\omega }-3/16{\left(\sum_{i=1}^{M}p\left(c_{i}\right)\left({\left(w^{T}\sum_{c_{i}}w\right)}^{2}-1\right)\right)}^{2}$
(3) Choose the *L* columns of *W* with highest mutual information
(4) Acquire the raw channel number of the *L* columns of *W* with highest mutual information

*Output*: preprocessing matrix *W* and channel number with highest mutual information

## Data Availability

The data used to support the findings of this study are available from the corresponding author upon request.

## References

[1] Kuiken T. A., Li G., Lock B. A. (2009). Targeted muscles reinnervation for real-time myoelectric control of multifunction artificial arms. *JAMA*.

[2] Li X., Chen S., Zhang H. (2016). Towards reducing the impacts of unwanted movements on identification of motion intentions. *Journal of Electromyography and Kinesiology*.

[3] Nishikawa D. (1999). EMG prosthetic hand controller using real-time learning method. *IEEE International Conference on Systems, Man, and Cybernetics*.

[4] Dipietro L., Ferraro M., Palazzolo J. J. (2005). Customized interactive robotic treatment for stroke: EMG-triggered therapy. *IEEE Transactions on Neural Systems and Rehabilitation Engineering*.

[5] Li G., Li Y., Yu L. (2011). Conditioning and sampling issues of EMG signals in motion recognition of multifunctional myoelectric prostheses. *Annals of Biomedical Engineering*.

[6] Zhang X., Zhou P. (2014). Myoelectric pattern identification of stroke survivors using multivariate empirical mode decomposition. *Journal of Healthcare Engineering*.

[7] Englehart K., Hudgins B. (2003). A robust, real-time control scheme for multifunction myoelectric control. *IEEE Transactions on Biomedical Engineering*.

[8] Adewuyi A. A., Hargrove L. J., Kuiken T. A. (2015). An analysis of intrinsic and extrinsic HandMuscle EMG for improved pattern recognition control. *IEEE Transactions on Neural Systems and Rehabilitation Engineering*.

[9] Xie H., Huang H., Wu J. (2015). A comparative study of surface EMG classification by fuzzy relevance vector machine and fuzzy support vector machine. *Physiological Measurement*.

[10] Rd W. T. (1990). Practical methods for controlling powered upper-extremity prostheses. *Assistive Technology*.

[11] Hudgins B., Parker P., Scott R. N. (1993). A new strategy for multifunction myoelectric control. *IEEE Transactions on Biomedical Engineering*.

[12] Mesa I., Rubio A., Tubia I. (2014). Channel and feature selection for a surface electromyographic pattern recognition task. *Expert Systems with Applications*.

[13] Holtermann A., Roeleveld K., Karlsson J. S. (2005). Inhomogeneities in muscles activation reveal motor unit recruitment. *Journal of Electromyography and Kinesiology*.

[14] Monica R. M., Mañanas M. A., Alonso J. F. (2012). High-density surface EMG maps from upper-arm and forearm muscles. *Journal of NeuroEngineering and Rehabilitation*.

[15] Merletti R., Aventaggiato M., Botter A. (2010). Advances in surface EMG: recent progress in detection and processing techniques. *Critical Reviews in Biomedical Engineering*.

[16] Rojas M. M., Mañanas M. A., Alonso J. F. (2012). High-density surface EMG maps from upper-arm and forearm muscles. *Journal of NeuroEngineering and Rehabilitation*.

[17] Afsharipour B., Ullah K., Merletti R. (2015). Amplitude indicators and spatial aliasing in high density surface electromyography recordings. *Biomedical Signal Processing and Control*.

[18] Vieira T. M., Merletti R., Mesin L. (2010). Automatic segmentation of surface EMG images: improving the estimation of neuromuscular activity. *Journal of Biomechanics*.

[19] Huang H., Zhou P., Li G., Kuiken T. (2009). Spatial filtering improves EMG classification accuracy following targeted muscle reinnervation. *Annals of Biomedical Engineering*.

[20] Brunner C., Naeem M., Leeb R. (2007). Spatial filtering and selection of optimized components in four class motor imagery EEG data using independent components analysis. *Pattern Recognition Letters*.

[21] Ramoser H., Müller-Gerking J., Pfurtscheller G. (2000). Optimal spatial filtering of single trial EEG during imagined hand movement. *IEEE Transactions on Rehabilitation Engineering*.

[22] Wang D., Zhang X., Gao X. (2016). Wavelet packet feature assessment for high-density myoelectric pattern recognition and channel selection toward stroke rehabilitation. *Frontiers in Neurology*.

[23] Geng Y., Zhang X., Zhang Y. T. (2014). A novel channel selection method for multiple motion classification using high-density electromyography. *Biomedical Engineering*.

[24] Dornhege G., Blankertz B., Curio G. (2004). Boosting bit rates in noninvasive EEG single-trial classifications by feature combination and multiclass paradigms. *IEEE Transactions on Biomedical Engineering*.

[25] Zerby S. A., Herbison G. J., Marino R. J. (1994). Elbow extension using the anterior deltoids and the upper pectorals. *Muscles & Nerve*.

[26] Naik G. R., Baker K. G., Nguyen H. T. (2015). Dependence independence measure for posterior and anterior EMG sensors used in simple and complex finger flexion movements: evaluation using SDICA. *IEEE Journal of Biomedical & Health Informatics*.

[27] Negro F., Muceli S., Castronovo A. M., Holobar A., Farina D. (2016). Multi-channel intramuscular and surface EMG decomposition by convolutive blind source separation. *Journal of Neural Engineering*.

[28] Blankertz B., Tomioka R., Lemm S., Kawanabe M., Muller K. R. (2008). Optimizing spatial filters for robust EEG single-trial analysis. *IEEE Signal Processing Magazine*.

[29] Grosse-Wentrup M., Buss M. (2008). Multiclass common spatial patterns and information theoretic feature extraction. *IEEE Transactions on Biomedical Engineering*.

[30] Parra L., Sajda P. (2003). Blind source separation via generalized eigenvalue decomposition. *Journal of Machine Learning Research*.

